# Intelligent Financial Auditing Model Based on Deep Learning

**DOI:** 10.1155/2022/8282854

**Published:** 2022-08-28

**Authors:** Xiaofeng Dai, Weidong Zhu

**Affiliations:** ^1^Department of Engineering Management, Anhui Audit College, Hefei 230601, China; ^2^School of Management, Hefei University of Technology, Hefei 230009, China

## Abstract

The entire auditing process is complicated and tedious and requires a lot of human resources. Therefore, the intelligent development of auditing is the general trend. In order to improve the audit quality, this paper establishes an intelligent financial audit model that can predict the audit opinion of the consolidated financial statements. This paper proposes an audit opinion prediction model based on the fusion of deep belief neural network (DBN) and long-short term memory (LSTM). First, an indicator system is established for audit opinions, and multiple financial parameters are used to describe possible audit opinions. On this basis, a DBN network is designed to complete deep feature extraction and used for LSTM training. According to the prediction model obtained by training, the subsequent audit opinion can be scientifically predicted. In the experiment, the method in this paper is tested based on financial audit related data sets and compared with the prediction results of traditional multilayer perceptron (MLP), convolutional neural network (CNN), and LSTM models. The results verify the validity and reliability of the model in this paper.

## 1. Introduction

As an external corporate governance mechanism, auditing plays an important role. The governance effect of auditing is directly reflected in the quality of auditing. The overall objective of an audit is to obtain reasonable assurance that the financial statements are free from material misstatement due to fraud or error. It aims to issue an audit report in accordance with auditing standards and to communicate with the client's management [1–3]. To achieve these goals, under the modern risk-oriented audit model, the main line of audit work requires auditors to identify, evaluate, and respond to the risks of material misstatement. Consistent with audit objectives, audit quality refers to the joint probability that auditors detect and report material misstatements. The realization process of audit quality can be summarized as finding, adjusting, and reporting material misstatements to achieve audit quality. How to achieve audit objectives and improve audit quality has always been the focus of audit research.

In the above context, many scholars have established models for predicting audit opinions and used these models to plan audit procedures. It was used as a quality control tool in the commitment review stage and to analyze variables that affect the probability of obtaining a qualified opinion. Reference [4] constructed a multicategory audit opinion prediction model based on the back propagation (BP) neural network method and tested it. Reference [5] used multiple financial indicators as eigenvalues of modeling data for the four types of audit opinions issued by companies and established a multicategory audit opinion prediction model based on error correction output coding and support vector machine (SVM). Reference [6] established a two-category prediction model of bank loan risk level classification authenticity audit based on SVM. However, most models for forecasting audit opinions have only been developed in the context of individual financial statements, and none of the models dealt with consolidated financial statements. In recent years, the rapid development of deep learning algorithms has provided a good tool for data prediction. Deep learning models such as multilayer perceptron (MLP), convolutional neural network (CNN), deep belief neural network (DBN), and long-short term memory (LSTM) have been widely used and verified in various aspects such as traffic flow, enterprise risk, equipment life, and so on [7–12]. In the field of financial auditing, the continuous application of new models and algorithms to improve forecast accuracy is an important aspect in the future.

Based on the existing literature, this paper designs a model that can predict audit opinions on consolidated financial statements based on a deep learning model. The proposed method combines DBN and LSTM. Among them, DBN is mainly used for deep feature learning to extract discriminative features from massive financial design data. On this basis, the LSTM is trained through the extracted features to build a prediction model. In the experiment, verification is carried out based on real corporate financial data. The samples were divided into the unqualified opinion group and the qualified opinion group during model training and provided a set of initial explanatory variables for the consolidated financial statements. These variables include financial parameters (efficiency, liquidity, profitability, solvency, productivity, and scale), corporate governance measures, and other qualitative parameters. After experimental verification, the method in this paper has performance advantages compared with several existing prediction methods.

## 2. Deep Learning Models and Prediction Algorithms

### 2.1. LSTM

LSTM is a variant of the traditional recurrent neural network (RNN). Since RNN is trained by time series gradient descent, the network may experience the problem of gradient disappearance or gradient explosion when the sequence is long and the feedback adjustment is performed. To overcome this problem, researchers proposed to use LSTM gating units to replace RNN units, making the network robust to prevent gradient vanishing (and exploding). So, the modified networks are suitable for training and classifying long time series [13–15].

Figure 1 shows the basic LSTM unit structure. The key to LSTM is the state of the cell *C*_*t*_. In order to add or delete the information in the cell, 3 gates are used in LSTM to control the training, namely the forgetting gate, the input gate, and the output gate. The gate determines the way the information passes through and protects and controls the cell state.

The forget gate uses a sigmoid layer to determine the information to be deleted in the cell state, which is calculated according to formula (1). For the input *x*_*t*_ and *h*_*t*−1_, the forget gate will output a number in the range [0, 1] and put it into the cell state *C*_*t*−1_. When it is 0, all are deleted; when it is 1, all are retained.

(1) $$\begin{array}{c} f_{t}=\sigma \left(W_{f}\cdot \left[h_{t-1},x_{t}\right]+b_{f}\right). \end{array}$$

In equation (1), *x*_*t*_ is the input at time *t*; *h*_*t*_ is the hidden layer state at time *t*; *f*_*t*_ is the output state of the forget gate at time *t*; *σ* is the sigmoid activation function; *W*_*f*_ is the weight matrix; *b*_*f*_ is the bias vector. The process of adding new information to a cell can be divided into two steps. First, LSTM uses an input gate containing a sigmoid layer to determine which information should be retained. The calculation process is represented by equation (2). Second, it uses a tanh function to generate a vector for these information, which is used to update the cell state ${\tilde{C}}_{t}$. The calculation process is represented by equation (3).

(2) $$\begin{array}{c} i_{t}=\sigma \left(W_{i}\cdot \left[h_{t-1},x_{t}\right]+b_{i}\right), \end{array}$$

(3) $$\begin{array}{c} {\tilde{C}}_{t}=\tanh\left(W_{C}\cdot \left[h_{t-1},x_{t}\right]+b_{C}\right). \end{array}$$

On the basis of the forget gate and the input gate, the cell state can be updated according to the following equation:

(4) $$\begin{array}{c} C_{t}=f_{t}\cdot C_{t-1}+i_{t}\cdot {\tilde{C}}_{t}, \end{array}$$

where *f*_*t*_*·C*_*t*−1_ indicates the information to be deleted; $i_{t}\cdot {\tilde{C}}_{t}$ refers to the newly added information.

The output gate determines the output content of LSTM, and the calculation is shown in equations (5) and (6). First, the sigmoid function is used to determine the cell content to be output, and then the tanh function is used to convert the cell state value between −1 and 1 to obtain the final output:

(5) $$\begin{array}{c} O_{t}=\sigma \left(W_{o}\cdot \left[h_{t-1},x_{t}\right]+b_{O}\right), \end{array}$$

(6) $$\begin{array}{c} h_{t}=O_{t}\times \;\tanh\;C_{t}. \end{array}$$

After the forward propagation, the output of the LSTM is connected to the fully connected layer, and the softmax classifier is used for processing to obtain the corresponding prediction result.

### 2.2. DBN

A multilayer restricted Boltzmann machine (RBM) is a neuroperceptron [16]. It [17] consists of an explicit layer and a hidden layer. The neurons in the two-layer structure are binary units, and the value of each neuron is 0 or 1. The RBM of each layer is through the contrastive divergence (CD) algorithm to achieve fast training. The basic structure of RBM is shown in Figure 2.

In the figure, *v* represents the visible layer; *h* represents the hidden layer; *w* is the connection weight between the visible layer and the hidden layer; *a* is the bias vector of the visible layer.

The energy function of RBM can be expressed as

(7) $$\begin{array}{c} E\left(v,h\right)=-\sum_{i=1}^{n}b_{i}v_{i}-\sum_{j=1}^{m}c_{j}h_{j}-\sum_{i=1}^{n}\sum_{j=1}^{m}w_{ij}v_{i}h_{j}. \end{array}$$

Accordingly, in a layer of RBM, the probability of the hidden layer neurons being activated is

(8) $$\begin{array}{c} P\left(h_{i}|v\right)=\sigma \left(b_{i}+\sum_{i}w_{ij}v_{i}\right). \end{array}$$

The core of DBN is composed of multilayer RBM and one-layer back-propagation neural network [18–20]. Among them, the core function of RBM is to do unsupervised learning. Through recursive RBM, the characteristics of information can be reflected in various types of sample spaces. RBM sets the feature factors that have been trained as the input, uses parameters, adjusts the network layer by layer, and finally realizes the prediction of the model. DBN consists of the input layer, hidden layer, and output layer. When building a DBN model, it is first necessary to determine the number of hidden layers, the number of nodes in each hidden layer, batch size, learning rate, and momentum. The hidden layer of the DBN is composed of several RBM stacks, and the data are extracted layer by layer through the RBM to obtain the abstract high-level features of the input data. Finally, the fault is classified by softmax.

### 2.3. Financial Audit Forecast Model Construction and Evaluation

In view of the complexity of financial audit data, this paper adopts several representative parameters to characterize, mainly including financial parameters, nonfinancial parameters, and other qualitative parameters including the liquidity, efficiency, solvency, productivity, and scale parameter. On this basis, the deep learning model is used for processing and prediction. In this paper, an audit model based on DBN-LSTM is constructed, which makes full use of the advantages of the DBN multilayer perceptron structure. It can better retain the attributes of the original data and solves the problem of feature extraction of financial audit data, thereby improving the prediction accuracy.  Figure 3 shows the basic flow of the model in this paper, and the specific implementation steps are as follows:

  Step 1. Data preprocessing. The original financial audit data are preprocessed, and singular value points and invalid data are proposed.
  Step 2. Deep feature extraction. The DBN network is trained to extract the deep features of the financial audit data and complete the unsupervised learning training process.
  Step 3. Training phase. The deep features extracted by the optimized DBN are input into the LSTM network, and a prediction model is established after training.
  Step 4. Testing phase. The divided test set is input into the trained prediction model to obtain the predicted value of the financial audit result.

In order to verify whether the prediction results of the model are true and reliable, this paper defines the evaluation indicators for quantitative calculation. Assuming that the predicted value and the actual value are divided by $\hat{y}=\left\{{\hat{y}}_{1},{\hat{y}}_{2},\ldots ,{\hat{y}}_{n}\right\}$ and *y*={*y*_1_, *y*_2_,…, *y*_*n*_}, the root mean square error (RMSE) and mean absolute percentage error (MAPE) are selected as the evaluation indicators of model accuracy. The expressions of them are as shown in equations (9) and (10):

(9) $$\begin{array}{c} \text{RMSE}=\sqrt{\frac{1}{n}\sum_{i=1}^{n}{\left({\hat{y}}_{i}-y_{i}\right)}^{2}}, \end{array}$$

(10) $$\begin{array}{c} \text{MAPE}=\frac{1}{n}\sum_{i=1}^{n}\left|\frac{\left({\hat{y}}_{i}-y_{i}\right)}{y_{i}}\right|\times 100\%. \end{array}$$

Accordingly, the smaller the RMSE and MAPE values are, the closer the predicted value is to the real value, and the higher the prediction accuracy is.

## 3. Experiment and Analysis

### 3.1. Dataset

To verify the performance of our method in predicting financial audit opinions, we randomly select 350 companies operating in Beijing in 2021. The audit opinions and group financial information in the sample are obtained from the Internet. Audit opinions are roughly divided into two categories. One is the report with unqualified opinion, that is, the report that fully complies with accounting standards. The other is the report with qualified opinion, that is, the report that does not comply with accounting standards. 125 financial statements received qualified opinions, and 225 financial statements received unqualified opinions. According to the statistical results, compared with the group with unqualified opinions, the group with qualified opinions has poorer results in terms of financial variables, that is, the level of profitability, liquidity, solvency, and productivity of companies with qualified audit opinion is lower. Therefore, the experimental results are in line with the actual situation.

In order to evaluate the performance of the proposed model, taking into account that the number of samples is not very large, a five-fold cross-validation process repeated 100 times is used in the experiment. For each of these 100 tests, the modes of training, validation, and testing are randomly selected, and all passed the model training and evaluation.

### 3.2. Results and Analysis

In order to test the pros and cons of the performance of the proposed method, three existing prediction models are selected for simultaneous comparison experiments, i.e., MLP, CNN, and LSTM. Among them, the LSTM method in the comparison method directly trains and predicts, and there is no DBN in this method.  Table 1 shows the test results of various methods under the two evaluation indicators. It can be seen that the method in this paper can achieve the best performance under both conditions, showing its effectiveness. In particular, compared with the LSTM method, the performance improvement of our method mainly benefits from the deep feature learning of DBN. Therefore, the DBN-LSTM method proposed in this paper has stronger adaptability to financial audit forecasting.

Considering the influence of noise and interference in the data, this paper adds different degrees of noises to the sample set according to the definition of signal-to-noise ratio (SNR). On this basis, a retest is carried out according to the above ideas, and the statistical results are shown in Table 2 using RMSE as the evaluation index. It can be seen that even in the case of strong noise interference, the method in this paper can still maintain a strong performance advantage, which further reflects its effectiveness.

## 4. In Conclusion

This paper studies the audit opinion prediction model and consolidated financial statements. On this basis, it introduces the methods, samples, variables, and main results of audit opinion prediction and proposes an audit prediction model combining DBN and LSTM. The proposed method effectively combines the advantages of DBN in deep feature extraction and the characteristics of LSTM in processing time series, which improves the accuracy of audit opinion prediction. In the experiment, the proposed method is tested based on financial audit-related data and compared with several existing data prediction models. The results reflect the performance advantages of this method. The effective application of the method in this paper can reduce the computational overhead of audit data analysis, thereby improving the accuracy and efficiency of audit analysis.

## Figures and Tables

**Figure 1:** Basic structure of LSTM.

**Figure 2:** Basic structure of RBM.

**Figure 3:** Basic procedure of the proposed method.

**Table 1:** Comparison of performance of the different methods using RMSE and MAPE.

Method	RMSE	MAPE (%)
Proposed	201.3	67.2
MLP	256.1	79.3
CNN	221.4	74.3
LSTM	219.3	71.2

**Table 2:** Comparison of performance of different methods under noises using RMSE.

Method	SNR (dB)			
	−10	−5	0	5
Proposed	302.1	267.3	232.1	211.5
MLP	330.9	312.3	296.4	274.1
CNN	318.1	282.1	261.2	231.4
LSTM	314.7	279.9	243.8	228.1

## Data Availability

The dataset can be accessed upon request.
